# Automated Detection of Nonmelanoma Skin Cancer Based on Deep Convolutional Neural Network

**DOI:** 10.1155/2022/6952304

**Published:** 2022-02-10

**Authors:** Muhammad Arif, Felix M. Philip, F. Ajesh, Diana Izdrui, Maria Daniela Craciun, Oana Geman

**Affiliations:** ^1^Department of Computer Science and IT, University of Lahore, Lahore, Pakistan; ^2^Department of Computer Science and Information Technology, JAIN (Deemed-to-be University), Kochi, Kerala, India; ^3^Department of Computer Science and Engineering, Sree Buddha College of Engineering, Alappuzha, Kerala, India; ^4^Stefan cel Mare University of Suceava, Suceava, Romania

## Abstract

One of the deadliest diseases is skin cancer, especially melanoma. The high resemblance between different skin lesions such as melanoma and nevus in the skin colour images increases the complexity of identification and diagnosis. An efficient automated early detection system for skin cancer detection is essential in order to save human lives, time, and effort. In this article, an automatic skin lesion classification system using a pretrained deep learning network and transfer learning was proposed. Here, diagnosing melanoma in premature stages, a detection system has been designed which contains the following digital image processing techniques. First, dermoscopy images of skin were taken and this is subjected to a preprocessing step for noise removal and postprocessing step for image enhancement. Then the processed image undergoes image segmentation using k-means and modified k-means clustering. Second, using feature extraction technology, Gray Level Co-occurrence Matrix, and first order statistics, characteristics are extracted. Features are selected on the basis of Harris Hawks optimization (HHO). Finally, various classifiers are used for predicting the stages and efficiency of the proposed work. Measures of well-known quantities, sensitivity, precision, accuracy, and specificity are used in assessing the efficiency of the suggested method, where higher values were obtained. Compared to the current methods, it is found that the classification rate exceeded the output of the current approaches in the performance of the proposed approach.

## 1. Introduction

One of the deadliest diseases that currently afflict humankind is cancer. Skin cancer is one of the most common and the deadliest among all types of cancer. Among these, melanoma is the most aggressive and deadly form [1] of cancer. Skin cancer are of two major sorts, namely nonmelanoma and melanoma (Merkel cell carcinomas, squamous cell, basal cell, and so on) [2] as shown in Figure 1. Melanoma is the dangerous skin cancer, however, if it is detected in the early stages, it can be curable, but progressive melanoma is deadly. Therefore, it is well known that the early treatment and detection of skin cancer can minimize the morbidity.

Additionally, the rate of unwanted biopsies is very high. The skin cancer image processing system used in diagnostics or diagnosis is the procedure of recognizing a skin texture or tissue by symptoms, signs, and the various kinds of diagnosis process results. Skin cancer is a malignant tumour located in the cells of the skin that is responsible for more than 50% of all cancers. Fortunately, skin cancer (squamous cell and basal cell, melanoma and malignant) is rare in children. When melanomas occur, they normally arise from pigmented nevi (moles) which are (diameter <6 mm) asymmetric, with irregular coloration and borders. A mass, itching, bleeding under the skin are other signs of cancerous change. The skin cancer detection system is the basic process to recognize and identify skin cancer diagnosis and symptoms in the early stages. The skin cancer detection system will be used to diagnose the skin cancer in the accurate stage [3, 4].

## 2. Related Work

Numerous studies in dermoscopic images have been conducted to identify skin lesions, but availability of classification using general images is very little. Esteva et al. [5] discussed the field of skin lesions classification into several groups. They grouped them into 23 separate categories of lesions. To conduct this classification, they used convolutional neural network (CNN) and used the 16-layer model VGG-16 and 19 layer model VGG-19 [6] generated by the Visual Geometry Group. Esteva et al. used VGG model that is pretrained and, with the assistance of transfer learning, enhanced its efficiency. The accuracy rate of 90% is obtained during classification of lesions.

Masood et al. [8] proposed an artificial neural network (ANN) system and classified cancerous and noncancerous lesions from 135 images. Using FCM Algorithm for Level Set Initialization, they divided images. They obtained the characteristics of images using histogram feature extraction method and statistical features by using the Gray Level Co-occurrence Matrix (GLCM). The three training algorithms used are Levenberg-Marquardt, Scaled-Conjugate Gradient, and Resilient Back Propagation, and a two-layer feed forward neural network is being trained. Using the Scaled Conjugate Gradient training algorithm, they achieved an accuracy of 91.9%. Zhang et al. [8] have examined the diagnosis of skin lesions. CNN for automatic recognition of skin cancer was considered in the study, contrasting this with other research methods. With a sensitivity of 95.00 % and specificity of 91.00 %, the proposed method attained a precision of 91.00 %.

The cutting-edge methods stated in the literature were reviewed by Pathan et al. [9], summarising these techniques. The steps involved are preprocessing of dermoscopic images, segmentation of these images, and extraction and collection of important characteristics and skin lesion disposition. Further, the analysis also assessed the implications of the methodologies mentioned in the literature. The Otsu threshold with active contour using a sparse-field level-set approach was the best result from the methods and algorithms mentioned, with a 97.50 % accuracy capacity for melanoma detection.

Using fine-tuned neural networks, Lee et al. [10] suggested the skin disease classification approach. In the validation set, an accuracy of 89.90% was obtained and in the evaluation set, the model obtained an accuracy of 78.50%. Harangi [11] attained the classification results in three groups of injuries making use of the technique of incorporating robust CNNs into a structure. The testing findings showed that in the process of categorising the 3 classes, the average area under receiver operating characteristic curve (AUC) was 89.10%.

Li and Shen [12] suggested two deep learning strategies for addressing 3 key tasks emerging in the field of image processing of skin lesions, i.e., segmentation of lesions (task 1), extraction of dermoscopic lesions (task 2), and classification of lesions (task 3). On the ISIC 2017 dataset, the proposed deep learning frameworks have been analysed. Experimental findings indicate that these constructs are promisingly accurate, i.e., 75.30% for task 1, 84.79% for the second task, and 91.20% for the third task. Ansari [13] suggested early detection of skin cancer using SVM. The dermoscopy images were collected and sent to various preprocessing techniques using filtering images. The unique highlights were picked using GLCM method and these were then used to define the classifier on the image and the accuracy obtained is about 95.00%.

Alcon et al. have developed a decision support system which takes image processing techniques for skin lesion assessment [14]. This also utilizes some patient history data before the diagnosis is made. An automatic classification system consisting of preprocessing, segmentation, and feature extraction steps was proposed by Cavalcanti et al. A two-stage classifier was proposed to recheck lesions labelled as benign [11] for reducing the missing rate of melanoma cases. Works [10, 11] seek to approximate the four ABCD rule requirements by obtaining a range of low-level characteristics. A collection of high-level characters that instinctively explain the ABCD rules [12] was suggested by Amelard. To enhance the quality of the image, a computer-aided system for preprocessing [13] was proposed by Giotis et al. Then, some of the lesions colour and texture properties are eliminated automatically. Afterwards, final decision is made by combining the physician decision based on physical examination and the output result developed by the CAD system [14, 15].

Deep learning techniques have also shown impressive outcomes in some areas like speech recognition, natural language processing [16, 17], computer vision areas such as object detection [18], object tracking [19, 20], and classification of images [20–24]. Without the need to collect handcrafted features, deep learning mechanisms achieve high precision for image classification. There seems to be a development in medical imaging activities, in particular, to take advantage of the greater potential of deep learning techniques [25–27]. CNN is a type of deep learning system where the raw image data are applied with trainable filters and pooling operations, automatically extracting a collection of complex high-level features [17–41].

### 2.1. Problem Statement

In order to prevent these debilitating treatments and obtain effective treatment, melanoma treatment includes chemotherapy and radiotherapy. Early diagnosis is among the most efficient solutions. For the identification of pigment skin lesions, several CAD systems are currently available, such as Dell'Eva-Burroni Melanoma Image Processing Software, which gives low performance in real implementations. However, general conclusions about the performance of these systems are hard to define. In organised research, the multiple image acquisition techniques such as dermoscopic, clinical, and normal camera images further complicate the classification task in one global methodology. Therefore, the new CAD programmes are also far from ideal and require further advances to enhance melanoma detection and diagnosis. In addition, two major problems are posed in the classification of skin pigment lesions into malignant and benign cancer.

- First, accurate segmentation is the difficult task to enhance the identification of abnormal lesions and the classification of these lesions into benign and malignant
- Second is the extraction of the most discriminatory set of characteristics that define the related features differentiating the pigment lesions into benign and malignant skin cancer

We plan to use deep learning techniques in this paper to form an automated diagnostic method for the detection of melanoma. The input images, normally exposed to lighting effects and the noise, are preprocessed for this purpose. As a result, this preprocessing lets CNN remove racist characteristics from the images. Then, to identify the input as melanoma or benign, the preprocessed images are given to the CNN architecture. Some methods, such as augmentation of dataset images, and the number of samples are increased to overcome the constraints of the training sample and the smaller number of images. Experimental analysis gives us a clear picture about the novelty of the proposed system with the existing methods.

## 3. Methodology

As for a proper diagnosis, the CAD systems provide a computer output to support analysis of radiologists to increase diagnostic accuracy and decrease the time to read the image. For early detection and diagnosis, the CAD method is also being explored. A CAD method is used for various images of tumours, such as dermoscopy, MRI, mammograms, and radiography. Five key stages from image acquisition to classification and diagnosis are used in the CAD system used in medical imaging such as data acquisition, preprocessing, segmentation, extraction of features and selection of features and, ultimately, classification. Each module is explained in detail in the later section of this proposal.

### 3.1. Dermoscopic Imaging and Skin Cancer

Dermoscopy, also named as Epi Luminescence Microscopy (ELM), is one of the most used noninvasive methods for the analysis of melanocytic and skin lesions that are pigmented. A portable, illuminated microscope called a dermatoscope is used to conduct this operation and is placed to the surface of the skin. This optical device consists of a 10-fold magnified, high-quality lens, a light source that is nonpolarized, a translucent plate, and a liquid medium between both the instrument and the skin. It enables skin lesions to be examined, unhindered by skin surface reflection, and is used for the histological and clinical correlation of lesions as shown in Figure 2. Dermoscopy significantly improves the diagnostic accuracy of melanoma, allows in vivo evaluation of colours, and enables the visualization of submacroscopical structures. It evaluates features such as pigment distribution and vascularization patterns and helps develop regression structures invisible to the naked eye.

#### 3.1.1. Datasets

In this work, mainly two different datasets are used: the dataset associated with the interactive Atlas of dermoscopy (EDRA) [28] and the recently proposed dataset from the International Skin Imaging Collaboration (ISIC), 2017 [8]. The dataset used in this work has around 2000 images for training, of which less than 400 are labelled as melanoma. It also includes 150 images and a set of 600 images as validation set that serve as test set. ISIC also provides segmentation masks for every image in the dataset, which classifies each pixel as belonging to the lesion or healthy skin. The EDRA dataset is smaller in comparison to ISIC; a subset of around 800 images will be used, of which around 240 correspond to melanomas. The exact numbers of images and their division between melanoma and nonmelanoma are presented in Tables 1 and 2.

### 3.2. Data Augmentation and Pre- and Postprocessing Operation

It is much difficult for an image to be processed and before getting processed, it needs to ensure that unnecessary items are removed from that image and then it successfully processed. In 2018, put forwarded enhancement methods for astrocytoma which brings various techniques such as histogram equalization for better preprocessing technique that can be used in MRI images of skin tumour. In 2013, Sudipta Roy brings out various preprocessing techniques in order to preprocess medical images of skin tumour such as median filter, low pass filter, and high pass filter. So, here for that CLAHE is put forwarded for discussion. After that, postprocessing is done, to remove the noise, thin hair, thick hair, and bubbles in the image. Here top-hat transformation and ADF-USM are used. ADF-USM filter performs pre- and postprocessing operation.

#### 3.2.1. Preprocessing by CLAHE

CLAHE is mainly used to evade noise amplification; here the algorithm is spited into small pre- and postimage forms called tiles. Until the required histogram is achieved, every single tile is been enhanced in separate manner [29]. Either Rayleigh or exponential are the parameters of histogram. The part where it is amplified in order to restrict contrast is done to avoid the amplification of noise. Another parameter called Clip-limit is used to restrict amplification by clipping histogram and thereby this method gives out better performance on before and after images [30, 31]. The algorithm of CLAHE is as follows:

(i) Input images, pre- and postmedical images of meningioma, are divided into subimages
(ii) Apply the following steps on each subimage:
  1. should obtain the highest value and histogram of subimage
  2. Repeat steps (a) and (b) to obtain histogram of subimage
  3. If the value of the required clip is lower than the bin value of histogram, then using that clip value clips that histogram
  4. For the value of bin going beyond the clip value given, there is a need to calculate the number of pixels
(iii) For each histogram bins, uniformly distribute the pixel that we calculated in order to obtain normalized histogram
(iv) Then get CDF values and, for every pixel in the image given, we need to find neighbouring pixels
(v) With the help of intensity of pixel values, based on the CDF values, gained mapping of neighbouring pixels has taken place
(vi) Within the range of [0-L-1], the pixels which are obtained are mapped under the new intensity values

#### 3.2.2. Adaptive Diffusion Filter Unsharp Masking

Anisotropic diffusion filter (ADF) is a nonlinear, space-variant transformation of the actual image. It is a very effective machine learning platform for image enhancement without supervision. Not only does it smooth the picture, but some important features such as the edges and textures are also preserved.

The filter unsharp mask (USM) is a simple method used by several researchers to increase the acuteness of images that are presumed to have low sharpness. With the support of a scaling parameter, it enhances the edges by subtracting an unsharp image from its original equivalent [32]. In several areas related to photography, this filter is used to improve the apparent resolution of fuzzy images. Inside the USM filter, the output of the amended anisotropic diffusion filter is used

(1) $$\begin{array}{c} U_{i,j}=a_{i,j}+\lambda \left[a_{i,j}-G_{i,j}\right], \end{array}$$

where *a*_*i*,*j*_ represents the input image; *λ* represents a sharpening parameter which must satisfy (*λ* > 0), where a higher value provides a sharper result; *G*_*i*,*j*_represents image *a*_*i*,*j*_ filter by a low − pass Gaussian filter.

To enhance the shape and edges of images, postprocessing is done.

#### 3.2.3. Top-Hat Transform

Top-hat transformation is a power full tool for doing the mathematical morphology to extract small information and elements from present images. It is possible to break the top-hat transformation into two forms. There are two transformations that are making white top-hat and black top-hat. Some structuring components define the white top-hat transformation as relation between the input image and the input image opening. The relationship between the closing operation by SE and the input picture is the black top-hat transformation. In order to separate the thick hair from image, black top-hat transform is used. The black top-hat transformation uses the structuring element as disk and the radius of disk will be taken as 8. The top-hat transformation method is used for correcting the effect of nonuniform illumination of light object having a dark background. The images containing the elements and objects are transformed using black top-hat based on their structural elements and their surrounding appearance.

### 3.3. Segmentation

The most significant step and the critical stage for classification and diagnosis is the correct identification of the skin lesion border. In this study k-means and modified k-means clustering, algorithms were developed and applied.

#### 3.3.1. K-Means Clustering

Clustering is widely used analysis method in emergency areas. Objects having similar character are grouped and they will be different from other set of groups. According to this algorithm, defining the number of clusters is done initially (*k*) and along with that randomly choosing the k-cluster center [33]. For each cluster, center distance is calculated and Euclidean function can be used for distance calculation (Figure 7).

K-means is a generally utilized unsupervised technique which divides the image into *k* segments dependent on the mean of each segment. To begin with, information is partitioned into *k* groups and after that the mean for each cluster will be determined as shown in Figure 3. Each datum is put in the bunch which has the nearest division to the mean of group using the Euclidean partition. The info data are a vector and the yield is a *k* vector. In order to apply k-means on CT pictures which are two dimensional, pixels should be set in one vector [33].

**Algorithm 1 .**

Initially input (*k*, data)
(1) Prefer *k* arbitrary located in the input space
(2) Allocate the group focus *μ*_*j*_ to those positions
(3) For each *x*_*i*_∈ data
(a) Calculate the distance Dist (*x*_*i*_, *μ*_*j*_) for each *μ*_*j*_
(b) Allocate *x*_*i*_ to the group with the lowest space
(4) For each *μ*_*j*_ shift the location of *mj* to the average points in that group:
  (2) $$\begin{array}{c} \mu_{j}=\frac{1}{N_{j}}\sum_{I=1}^{N_{j}}x_{I}, \end{array}$$

where *k* is the bunch quantity, *N*_*j*_ is the amount of available information in a cluster *j*, and *mj* is the average of bunch *j* and various square errors which resolve the situation of the repeat circle as

(3) $$\begin{array}{c} \text{SSE}=\sum_{j=1}^{K}\sum_{i=1}^{n}\text{dist}{\left(x_{i},c_{j}\right)}^{2}. \end{array}$$

The main flaw of this method is the amount of clusters. The *k* value is selected and is used to divide the image. Another inconvenience is affectability to anomalies, commotions, and starting qualities. From the information vector, the underlying qualities are chosen arbitrarily. To improve the issue, a few refinements have been done on this calculation and an upgraded calculation has been introduced.

#### 3.3.2. Modified K-Means Clustering (MKC)

K-means brings out simple and efficient algorithm for detecting tumour, but it has a demerit which is unable of detection of tumour even in precise manner and especially in the case of malignancy. So MKC comes into play, it works in small datasets as well as large ones, and also it reduces noise thereby bringing more accuracy to cluster [34].

Algorithm of MKC

- With the help of *imread* function in MATLAB environment images are been read
- With the help of making form and applying form images are converted to *L∗a∗b* colour space
- For each step evaluate mean
- Using k-means clustering label, classify the colours
- With the help of cluster, segmented images are done by colour

### 3.4. Feature Extraction

Feature extraction by histogram method gives only local features, so in order to consider spatial features, we use co-occurrence matrix-based feature extraction. GLCM matrix shows the frequency value of the grey level in a specified spatiality with the grey level value of the region of interest. The number of rows and columns within GLCM matrix shows the grey level or pixel colour of the image surface value [14–16, 18, 19].

Texture feature computations utilize the GLCM to calculate the intensity variation of the pixel of interest. Their computation mainly depends on 2 parameters such as relative distance between the pixel paired and their relative orientation. GLCM contains fourteen features, of them the most commonly valued features are entropy, contrast, energy, inverse difference moment, correlation, sum, and information measures of correlation.

*Energy.* this statistic is also referred to as uniformity or second moment of angular moments and is defined as the sum of squared GLCM elements. This test the uniformity of textures, which is pixel pair duplication. In textures, it identifies abnormalities. A maximum value of one is reached by energy. Energy has a normalised range. The GLCM includes a large number of small entries with a less homogeneous image. A function that measures the total likelihood of having unique patterns of grey scale in the picture is described as
  (4) $$\begin{array}{c} \text{energy}=\sum_{i=0}^{N_{p-1}}\sum_{j=0}^{N_{p-1}}p^{2}\left(i,j\right). \end{array}$$
*Contrast.* using gray-level co-occurrence matrix, it measures local variations. This statistic calculates an image's spatial occurrence and is the GLCM moment of difference. It measures the amount of local variance that is occurring in the picture. It is defined as
  (5) $$\begin{array}{c} \text{contrast}=\sum_{i=0}^{N_{p-1}}\sum_{j=0}^{N_{p-1}}{\left(i-j\right)}^{2}p\left(i,j\right). \end{array}$$
*Correlation.* this measures the occurrence in the GLCM matrix of a joint likelihood of the defined pairs of pixels. Correlation shows how a pixel is correlated to its neighbour across an image, identified as an image
  (6) $$\begin{array}{c} \text{correlation}=\sum_{i=0}^{N_{p-1}}\sum_{j=0}^{N_{p-1}}\frac{\left(i-µ\right)\left(j-µ\right)p\left(i.j\right)}{\sigma_{i}\sigma_{j}}. \end{array}$$
*Homogeneity.* this is the estimation of a closeness of GLCM distribution elements to GLCM diagonal elements. The Inverse Difference Moment is often the technique. It measures image homogeneity, to small grey value variations; it expects higher values in some components. If all elements of the image are all the same, it has the maximum value. It is defined as
  (7) $$\begin{array}{c} \text{homogeneity}=\sum_{i=0}^{N_{p-1}}\sum_{j=0}^{N_{p-1}}\frac{p\left(i,j\right)}{1+\left|i-j\right|}. \end{array}$$

### 3.5. Histogram-Based (Statistical) Features

Colour features are mean, standard deviation, kurtosis, skewness, and entropy. Entropy provides the amount of image information that is needed for compression of image. These characteristics are extracted using the descriptor for colour moment (CM). Equations for statistical characteristics are given as

(8) $$\begin{array}{c} \text{mean}:\;\mu_{i}=\frac{1}{N}\sum_{j-1}^{N}f_{ij},\\ \text{SD}:\;\sigma_{i}={\left(\frac{1}{N}\sum_{j-1}^{N}{\left(f_{ij}-\mu_{i}\right)}^{2}\right)}^{1/2},\\ \text{skewness}:\;\gamma_{i}={\left(\frac{1}{N}\sum_{N}^{1}{\left(f_{ij}-\mu_{i}\right)}^{3}\right)}^{1/3},\\ \text{kurtosis}:\;\delta_{i}{\left(\frac{1}{N}\sum_{N}^{1}{\left(f_{ij}-\mu_{i}\right)}^{4}\right)}^{1/4},\\ \text{entropy}:\;\varepsilon_{i}=-\sum_{j-1}^{N}\left(f_{ij}*\;\log\;f_{ij}\right). \end{array}$$

## 4. Feature Selection

Not all the features make a payment to the classification process. Feature selection is carried out with the aim of identifying the most suitable feature set. Proposed system makes use of Improved HHO for selection [35].

The following are the steps in HHO algorithm:

1. By using a random function, the population *X* is initialized, where N is the size.
2. Best fittest solution N is calculated by applying the EOBL technique.
3. Use the HHO algorithm to adjust the location of each position in the population according to the best fitness value, using HHO algorithm and the Rabbit.
4. Use a mutation strategy for a good rabbit location. If the current location has a greater fitness value than the previous, then new location is considered to be future rabbit location, which has to be implemented using MNS strategy, which in turn can be used for further boosting of the location.
5. An iteration process is carried out and continues until the current rabbit position is matched to the potential rabbit location. If the current position of a rabbit is good than future location of the rabbit, then rollback strategy is introduced; otherwise, the position of the rabbit is changed to the future location of the rabbit.
6. The process is repeated till the termination criteria are reached.

### 4.1. Classification

In 2020, Hassan Ali Khan put forward his CNN model that gives greater accuracy and performance when compared to other neural networks in order to classify these skin tutor images. Milica brings out another version of CNN model which can be used for classifying these skin tumour images into three categories and gives 96.5% accuracy higher than other models. In this paper different neural networks such as Hybrid CNN-IHHO with ResNet, VGG, and DenseNet are discussed in order for the classification of melanoma images to reach the presence of normal and abnormal melanoma tumour, in which Hybrid CNN gives much improved performance in terms of accuracy than other methods.

#### 4.1.1. CNN Classifier

It is a difficult process to derive an efficient and discriminatory feature set that specifically differentiates between different classification groups. There is a pitfall that we can feed some inconsistent features to the network by using a wide collection of features. On the other hand, there is a probability that certain correct descriptors are lacking by using a limited collection of features. Therefore, without the need to specify handcrafted feature extraction procedures, automated feature extraction systems may be used to attain a discriminatory feature set on the basis of a branded training set. As a deep learning platform, CNN is used in this paper for automated melanoma detection. A series of efficient convolve-filters is used by CNNs. In input images, they are able to analyse different structures. Therefore, the image itself is the input when using CNN and the network itself collects suitable elements of the image. CNNs usually involve several layers of convolve and pooling, and a completely linked layer is made of the last layer. The convolve layer filters the input image with a kernel package where each convolution layer is normally followed by a pooling layer. The pooling layer lowers the dimension of the feature map in each given window by selecting the mean or maximum values. It is accomplished for the purpose of identifying the images with certain general patterns that are perceptible. In this article, CNNs consist of two converting layers with a 5 × 5 kernel. In the first convolution layer, there are twenty feature maps and in the second there are fifty feature maps [26–34, 36–38].

The convolutional layer contains a series of convolutional kernels in which each neuron behaves as a kernel. Here, the convolution operation changes to a correlation operation if the kernel is symmetric. By splitting the picture into small slices, generally known as receptive fields [32], the convolutional kernel works. The operation can be written as follows:

(9) $$\begin{array}{c} f_{1}^{k}\left(p,q\right)=\sum_{c}\sum_{x,y}i_{c}\left(x,y\right).e_{1}^{k}\left(u,v\right), \end{array}$$

where *i*_*c*_(*x*, *y*) is an element of *I*_*c*_, where *I*_*c*_ is the input image tensor, that is multiplied by *e*_1_^*k*^(*u*, *v*) index of the *k*^th^ convolutional kernel *k*_1_ of the *l*^th^ layer. The output feature-map of the *k*^th^ convolutional operation can be defined as

(10) $$\begin{array}{c} F_{1}^{k}=\left[f_{1}^{k}\left(1,1\right),\ldots \left(f_{1}^{k}\left(p,q\right),\ldots f_{1}^{k}\left(P,Q\right)\right)\right]. \end{array}$$

It combines similar data in the receptive field neighbourhood and generates the dominant outcome within this local area.

(11) $$\begin{array}{c} Z_{l}^{k}=g_{p}\left(F_{l}^{k}\right). \end{array}$$

Equation (11) gives the pooling operation where *Z*_*l*_^*k*^ denotes the pooled feature-map of *l*^th^ layer for *k*^th^ input feature-map *F*_*l*_^*k*^, whereas *g*_*p*_ (.) gives the pooling operation type. The use of pooling operation helps in extracting the features that are invariant to small distortions and translational shifts. The activation function is expressed in

(12) $$\begin{array}{c} T_{l}^{k}=g_{a}\left(F_{l}^{k}\right). \end{array}$$

Here, *F*_*l*_^*k*^ is the output that is given to the activation function *g*_*a*_ (.) and adds nonlinearity thus giving an output *T*_*l*_^*k*^ for *l*^th^ layer.

Following each convolution sheet, there is one pooling layer. The outputs are such that the 4 layers are transferred to a completely linked 2-layer stage with 100 and 2 neurons, respectively. With a linear transfer feature, this 2-layer network forms the final diagnostic results.

Batch normalization for a transformed feature-map *F*_*l*_^*k*^ is shown in

(13) $$\begin{array}{c} N_{l}^{k}=\frac{F_{l}^{k}-\mu_{B}}{\sqrt{\sigma_{B}^{2}+\varepsilon }}. \end{array}$$

In (13), *N*_*l*_^*k*^ represents normalised depict mean and *μ*_*B*_ and *σ*_*B*_^2^ feature-map, *F*_*l*_^*k*^ is the input feature-map, and B represents the variance of a feature-map for a small batch.

The CNN architecture of the proposed method is shown in Figure 4. The images of the sample are provided to the proposed CNN after removal of noise and illumination errors.

There should be a sufficient number of samples to adequately train every CNN. But, due to the problems in obtaining and marking images, there are generally small numbers of images present in datasets. We can, therefore, cope with the restricted training package. There are several automated techniques extending the training data for this reason. Taking an example case by cropping the image 5% from the top and 5% from the left side, it is cut from its top-left corner. The new picture would then be scaled down to the original size. This form of cropping can be performed from three other corners as well. This can be also done with 10% cropping. Besides the original image, this results in 8 pictures. The resultant 9 images were rotated by 0, 90, 180, and 270 degrees afterward. Furthermore, within each input images 36 synthetized images are extracted and the size of the training dataset will be multiplied by 36. The 188 × 188 pixels are resized for all input images. 36 versions of images were generated by cropping and rotation for testing data. By considering the results of its 36 synthesised versions, the final diagnosis is done.

#### 4.1.2. R-CNN

As an inspiration from VGG-19, the development of ResNet model occurred and it is one of the deepest architectures proposed. Size of the convolutional layers in this ResNet model is of 33 filters, and also the layers here all have the same filters as for output feature map and if the feature map is spited to half due to doubling of number of filters, that will be better for maintaining the time complexity of every layer [28, 38]. With the stride value of two, it executes the down sample. The termination of ResNet happens with SoftMax activated fully connected layer and global average pooling layer.

Figure 5 implies the residual learning interpretation as subtraction of input features which are learned from that layer. For that ResNet uses connections which are shortcut for each pair of 33 filters and inputs of *K*^th^ layer to (*K*+*x*)^th^ layer are connected. To avoid these vanishing gradients, issued layers are bypassed and activation layers are reutilized from the preceding layer to layer that is situated next to that which learned its weights. It was way simple and easier for training these networks than deep CNN because it resolves accuracy degradation. The ResNet used here is ResNet-101 and it contains 101-layer residual network and is the modified version of the 50 layered ResNet.

#### 4.1.3. VGG-CNN

So, here pretrain VGG-16 neural network and freeze some layers so that it is fine tuned in order to avoid overfitting issue due to small dataset [28]. VGG-16 is a 16-layer convolutional neural network and our image size is of 512 × 512, which basically includes 16 conv. layer of 3 × 3 filter and 5 Max pooling layers of size 2 × 2. On the top, there will be 2 fully connected layers along with a SoftMax output layer. Since this network is large and contains literally 138 million parameters, conv. layers are stacked in order to build deep CNN for improving in learning hidden features, Figure 6.

#### 4.1.4. D-CNN

One of the special cases of convolutional neural network is DenseNet, where the current layer is connected with the entire layer that is previously existed. The structure of this network brings some merits better than other networks such as in the case of vanishing gradients, feature propagation strengthening, reusing of features, and mostly reducing the number of parameters. Between each consecutive dense block, there is convolutional and pooling layers connected sequentially.

The preprocessed image is fed to feed forward network which literally connects each layer to every other layer; hence, it is a dense net. The preprocessed image is fed to convolution layer of 24-filter, each dense block contains dense connection of 6 layers, and this layer performs function like batch normalization, activation, and convolution. Activation function ReLU is used and with a 3 × 3 × 3 kernel 12 filters of convolutional layer are made. The transition block (conv. and pool layer) forms 1 × 1 × 1 convolution with no repetition. Thereby at final stage a SoftMax function is used for classifying meningioma tumour images.

In Figure 7 it shows the performance evaluation of different classification techniques such as VGG, ResNet, and DenseNet along with the methods that this paper put forwarded like Hybrid CNN classifier and thereby it is clear that CNN gives the highest accuracy out of all, i.e., 98% and the rest of the methods VGG with 95%, ResNet with 93.5%, and finally DenseNet with 86.7%.

#### 4.1.5. Improved HHO-Based CNN

Using feature vector, skin tumour is detected and segmented using HHO and the extracted features are sent to CNN for classification [39–41]. HHO is inspired from the obliging behaviour and style of chasing of Harris Hawks and this method was so efficient in giving solutions. It poses to tackle complex of search space while considering issues like deceptive optima, local optima, and multimodality. Performance of HHO yields better when WOA is incorporated and thereby control the convergence rate [13].

Harris Hawks optimization (HHO) is one of the most recent and mostly used gradient-free, optimization algorithms that mimic the Harris Hawks' birds' chasing style. Recently, Haidari et al. introduced HHO in 2019 [33]. This algorithm takes up the Harris Hawks attacking practices, such as predation, preaching, and surprise pounce tactics, on the prey in nature. HHO has got 2 main stages, like other metaheuristic algorithms: exploration and exploitation, but HHO has again got 2 phases for exploration and 4 phases for exploitation, which are defined as follows.

In certain conditions, the detection of target according to Harris Hawks depends on the following:

(14) $$\begin{array}{c} x\left(t+1\right)=\left\{\begin{array}{c} X_{\text{rand}}\left(t\right)-r_{1}\left|X_{\text{rand}}\left(t\right)-2r_{2}X\left(t\right)\right|Q\geq 0.5,\\ \left(X_{\text{rabbit}}\left(t\right)-X_{m}\left(t\right)\right)-r_{3}\left(LB+r_{4}\left(UB-LB\right)\right)Q\leq 0.5. \end{array}\right. \end{array}$$

Here, *x*(*t*+1) is the Hawks position in the coming iteration *t*, *X*_rabbit_(*t*) is the rabbit position, *x*(*t*) represent the Hawk's current position, and*X*_*m*_(*t*) gives the average position based on Hawk's population. *r*_1_, *r*_2_, *r*_3_, *r*_4_, and *q* (wait) are the variables that were randomly chosen numbers within the interval [0, 1], and the upper and lower bounds were represented by LB and UB. HHO mainly concentrates on the direct method to calculate the average position of Hawks *X*_*m*_(*t*) by

(15) $$\begin{array}{c} X_{m}\left(t\right)=\frac{1}{N}\sum_{i=1}^{N}X_{i}\left(t\right), \end{array}$$

where the position is represented by *X*_*i*_(*t*) in the iteration *t* and the Hawks total count is represented by *N*.

In HHO, the transition in between the exploration and exploitation phase, as well as between various exploitations phases, depends on the *E*, the prey escaping energy. HHO believes that the rabbit's energy decreases when escaping from the hawks, which can be measured as

(16) $$\begin{array}{c} E=E_{0}\left(1-\frac{t}{T}\right). \end{array}$$

Here *E* represents the escaping energy, *E*_0_ is the initial energy state that updates its value randomly over the interval (−1, 1), and *T* represents the maximum number of iterations. HHO redirects the hawks to explore various regions search for the rabbit when the escaping energy of the rabbit is |*E*| ≥ 1. But when the energy is reduced |*E*| < 1, during the exploitation process, the hawks check the neighbourhood for the solution.

HHO is built on the basis of four potential attack technique strategies. The *r* and |*E*| are the two variables that indicate which plan will be carried out. Although |*E*| is the rabbit's escape energy, *r* refers to the likelihood of escape, where *r* < 0 : 5 implies a greater chance of successful escape for the rabbit, and the failure to escape is referred by *r* ≥ 0 : 5.

The search ability of HHO is improved using EOBL technique. The opposition point is described as given: each *X*_*i*_=(*x*_*i*;1_; *x*_*i*;2_; …; *x*_*i*;*D*_) in the present population *X*_*e*_=(*x*_*e*;1_; *x*_*e*;2_; …; *x*_*e*;*D*_); then, the elite opposite point ${\overset{ˇ}{X}}_{i}=\left({\overset{ˇ}{x}}_{i;1};{\overset{ˇ}{x}}_{i;2};\ldots ;{\overset{ˇ}{x}}_{i;D}\right)$ can be mathematically expressed as

(17) $$\begin{array}{c} {\overset{ˇ}{x}}_{i;j}=s\times \left(da_{j}+db_{j}\right)-x_{i,j}, \end{array}$$

where *s* ∈ [*a*_*i*_, *b*_*i*_], *S* ∈ *U*[0,1]*S* is a generalized factor. *dl*_*j*_ and *dm*_*j*_ are known to be dynamic boundaries, that is expressed as

(18) $$\begin{array}{c} dl_{j}=\min\left(x_{i;j}\right),dm_{j}=\max\left(x_{i;j}\right). \end{array}$$

The corresponding opposite, however, will surpass the [*l*_*i*_, *m*_*i*_] search boundary. A random value within [*a*_*i*_, *b*_*i*_] is allocated to the transformed individual to solve this matter as follows:

(19) $$\begin{array}{c} {\overset{ˇ}{x}}_{i;j}=r\;\mathrm{and}\left(l_{j},m_{j}\right),\;\text{if}{\overset{ˇ}{x}}_{i;j}<l_{j}||{\overset{ˇ}{x}}_{i;j}>m_{j}. \end{array}$$

HHO value mainly depends on rabbit energy |*E*| to switch from phase to discovery to phase of exploitation and to select the new exploitation process. It also utilizes rabbit resources to stop the hawks from dropping into local optima.

Algorithm of IHHO-CNN

- First layer is applied with convolution filter
- Smoothening of convolutional filter is done for reducing the sensitivity of the filter and that is called subsampling
- Activation layer will control the transferring of signals between layers
- With the help of ReLU, training time is fastened
- Preceding layer neuron is connected to neurons in subsequent layer
- Loss layer is added as a feedback for neural network during training period
- Initializing parameters: related parameters are initialized
- (a) *A*={*A*1,…, *Af*}
- Error evaluation: on the basis of the fitness function, better solutions are obtained and that solution yields less MSE and MSE is calculated as follows: *MSerr*=1/*g*Σ*e*=1*g*[*Fg* − *Fg*′]2
- Weight update
- Error recomputation: errors are recalculated with the help of formula in fully connected layer and those generating less error are given to CNN training
- Optimum weights are determined: for each solution, errors are calculated and those having less errors are given to training process
- Termination

## 5. Experimental Results and Analysis

### 5.1. Performance Evaluation

The following equation gives the percentage of the actual lesion that is truly detected by the automated method. The performance metrics result of the proposed method is shown in (20).

Segmentation
  (20) $$\begin{array}{c} \text{Jaccard index}=J\left(c,d\right)=\frac{S\left(c\cap d\right)}{S\left(c\cup d\right)},\\ \text{dice overlap index}\left(\text{DOI}\right)=D\left(c,d\right)=2X\frac{c\cap d}{c+d},\\ \text{similarity index }\left(\text{SI}\right)=\frac{2\text{X true positive}}{2\text{X true positive}+\text{false positive}+\text{false negative}},\\ \text{absolute volume measurement error}\left(\text{AVME}\right)=\left(\frac{V_{\text{automatic}}}{V_{\text{manual}}}-1\right),\\ \text{figure of merit}\left(\varepsilon \right)=1-\left(\varepsilon \right)=1-\frac{\left|V_{\text{manual}}-V_{\text{automatic}}\right|}{V_{\text{manual}}}. \end{array}$$
Classification
  (21) $$\begin{array}{c} \text{sensitivity}=\frac{T_{r}\text{P}}{T_{r}\text{P}+F_{l}\text{N}}\times 100\%,\\ \text{specificity}=\frac{T_{r}\text{N}}{T_{r}\text{N}+F_{l}\text{P}}\times 100\%,\\ \text{accuracy}=\frac{T_{r}\text{P}+T_{r}\text{N}}{T_{r}\text{P}+F_{l}\text{P}+F_{l}\text{N}+T_{r}\text{N}}\times 100\%,\\ \text{precision}=\frac{T_{r}\text{P}}{T_{r}\text{P}+F_{l}\text{P}}\times 100\%,\\ \text{F}-\text{measure}=\frac{2*\text{precision}*\text{recall }}{\text{precision}+\text{recall }}. \end{array}$$

### 5.2. Simulation Environment

For the processing of medical image in image processing, MATLAB toolboxes have become a great resource for getting the accurate diagnostic result. The images can be processed and its selected features are analysed using the toolbox. If the classification algorithm mainly concentrates on neural network application, then this neural network toolbox can be used to build and train a neural network feed forward model used to classify these images into malignant groups and benign groups.

### 5.3. Experimental Results

For this classification techniques which are put forwarded and discussed, the following parameters such as accuracy, sensitivity, specificity, precision, and F1-score are evaluated. True positive (TP) offers the number of correctly identified cases, false positive (FP) provides wrongly identified cases, true negative (TN) provides safe cases, and eventually false negative (FN) results in good cases falsely identified. The resting parameters of the notes are defined as follows. 1. True positive: it gives the properly expected number of malignant lesions. 2. Positive: number of malignant lesions. 3. Real negative: the number of benign lesions that are accurately estimated. 4. Negative: the number of benign lesions shown. In Figures 8–10 the same operations will be followed. The input image is preprocessed (b & c) and then the colour image is converted to Gray scale image. For proper identification of skin texture, hairs in the skin are to be extracted, and for that top-hat transform is used. The image after hair removal is given into the ADF-USM to remove the noise. The image after noise removal is given to the unsharp masking to sharpen the image. Noise-and-hair-removed image is subjected to the k-means and modified k-means method to segment the image further decision taken on the basis of features extracted from the segmented image. Finally, display whether the image is benign, suspicious, or malignant.

The evaluation matrices are Dice coefficient, Jaccard index, accuracy, and MCC to find out the segmentation efficiency. The volume measurement of segmented ROI's and its ground truth values are shown in Table 3. The obtained result of Dice coefficient is an average of 0.80 and Jaccard index is 0.96. Each value shows betterment in the efficiency than modified k-means approach. Table 3 shows that modified k-means obtained good result than modified k-means method.

Statistical parameters are calculated by GLCM and FOS. The features values are shown in Table 4.

For each classifier that is given in Table 5, the accuracy is calculated in this work. The CNN + IHHO *r* yields the best results from the table relative to other classifiers. The contrast shows that the classifiers used in the present study clearly lead to better outcomes than other classifiers. Performance analysis of learning-based classifier is proposed for the diagnosis of melanoma cancer. It indicates that this is the best diagnostic technique for skin cancer.

## 6. Conclusion

So, this paper brings out a clear identification and classification of pre- and postcontrast melanoma skin tumour images and thereby shows the presence of benign and malignant meningiomas. The flow of steps contains preprocessing, segmentation, and classification in which each step results in different techniques analysed and discussed and also brings better evaluation. In the case of preprocessing, enhancement of images happen much in the case of CLAHE rather than in anisotropic diffusion filter. The modified *K*-means clustring provides better reuslts in group image segmentation as compared to other methods. These grouped images are given to classification part where these images are classified to produce result of malignant and benign melanoma tumours. For that various neural networks are discussed in which Hybrid CNN (CNN + IHHO) classifier gives much better accuracy than other methods like ResNet, VGG, and DenseNet. Finally, with the help of the above improved and evaluated methods we can easily identify and classify and most importantly diagnose them at early stages.

## Figures and Tables

**Figure 1:** Diagnosis trees structure for skin lesion.

**Figure 2:** Sample dermoscopic image from ISIC dataset.

**Figure 3:** Flowchart of k-means clustering.

**Figure 4:** CNN architecture.

**Figure 5:** A regular block (left) and a residual block (right).

**Figure 6:** VGG-16 networks.

**Figure 7:** DenseNet.

**Figure 8:** Benign sample: (a) input image, (b) contrast limited histogram equalization output, (c) ADF-USM, (d) Gray scale conversion, (e) contrast adjusted, (f) hair removal, (g) sharpening of image, (h) K-means clustering, and (i) modified K-means clustering.

**Figure 9:** Suspicious sample: (a) input image, (b) contrast limited histogram equalization output, (c) ADF-USM, (d) grey scale conversion, (e) contrast adjusted, (f) hair removal, (g) sharpening of image, (h) k-means clustering, and (i) modified k-means clustering.

**Figure 10:** Malignant sample: (a) input image, (b) contrast limited histogram equalization output, (c) ADF-USM, (d) grey scale conversion, (e) contrast adjusted, (f) hair removal, (g) sharpening of image, (h) k-means clustering, and (i) modified k-means clustering.

**Table 1:** ISIC-image distribution.

Subset	Melanoma	Nonmelanoma	Total
Train	254	654	908
Validation	25	112	137
Test	129	385	514

**Table 2:** EDRA-image distribution

Melanoma	Nonmelanoma	Total
231	359	590

**Table 3:** Segmentation results.

Methods		K-means	Modified k-means
Image 1	Dice Coefficient (DC)	0.9818	0.9863
	Jaccard coefficient (JC)	0.9642	0.9729
	MCC	0.9814	0.9859
	Accuracy	0.9991	0.9992

Image 2	Dice coefficient	0.7846	0.9133
	Jaccard coefficient	0.6456	0.8405
	MCC	0.7647	0.9163
	Accuracy	0.9989	0.9991

**Table 4:** GLCM and FOS features.

Image no.	GLCM feature				FOS feature				
	Contrast	Correlation	Energy	Homogeneity	Mean	Standard deviation	Skewness	Kurtosis	Entropy
1	0.008566	0.97740	0.6123	0.995717	0.006	0.01080	2.01778	6.76021	2.3850
2	0.005587	0.968634	0.8163	0.997207	0.013	0.018964	1.384442	3.37708	2.98339
3	0.005338	0.978297	0.7487	0.997331	0.009	0.012767	1.655632	4.73059	2.77234
4	0.005214	0.976312	0.7746	0.997393	0.011	0.013236	1.244131	3.33805	2.91287
5	0.006642	0.973369	0.7439	0.996679	0.011	0.019105	2.274177	7.10785	2.68715
6	0.005742	0.983522	0.6463	0.997129	0.006	0.010301	1.605176	4.28244	2.05357
7	0.008752	0.956693	0.7892	0.995624	0.008	0.010716	1.578003	4.13867	2.57759
8	0.004593	0.969224	0.8461	0.997703	0.010	0.01203	0.826578	2.47775	2.77483
9	0.009621	0.976871	0.5744	0.995189	0.011	0.01429	0.945757	2.65592	2.23901
10	0.00748	0.982728	0.5598	0.99626	0.010	0.008143	0.419944	2.28365	2.81441
11	0.0072	0.980558	0.6224	0.9964	0.014	0.01945	2.495946	12.0050	3.11189
12	0.00807	0.977549	0.6325	0.995965	0.012	0.01388	1.159288	3.16243	3.16398
13	0.00987	0.974196	0.6077	0.995065	0.014	0.02124	2.216729	9.24762	2.65219
14	0.013532	0.969236	0.5467	0.993234	0.008	0.010971	1.308686	4.27185	2.4252
15	0.013904	0.971696	0.4950	0.993048	0.009	0.013778	2.758114	11.6741	2.7070
16	0.015456	0.9312	0.7601	0.992272	0.009	0.010296	0.914299	2.52796	2.76609
17	0.009063	0.972961	0.6573	0.995469	0.006	0.01445	3.510672	15.6859	2.07587
18	0.011328	0.977156	0.4930	0.994336	0.011	0.019445	3.895612	19.3494	2.66697
19	0.009404	0.976413	0.5928	0.995298	0.008	0.021771	3.888284	17.3682	2.10227
20	0.003476	0.962276	0.9043	0.998262	0.016	0.023343	1.321097	3.09597	2.91838

**Table 5:** Performance metrics.

Classifier	Sensitivity	Specificity	Accuracy	Precision	Border error
CNN + IHHO	96.1	98.6	97.3	96	2.7
DCNN	98.5	90.66	94.6	91.35	5.4
VGG-CNN	92	92.4	94.7	89.3	5.3
RCNN	92.7	96	90	96.4	7.3
CNN	86.6	84	90	93.3	10
ANN	80.5	67	74	71.6	26
SVM	85	71.5	78	75	22

## Data Availability

The data supporting this study are from previously reported studies and datasets, which have been cited. The processed data are available upon request from the corresponding author.

## Abbreviations

BRATS: The Multimodal Skin Tumour Image Segmentation Benchmark
MRI: Magnetic resonance imaging
HCNN: Hybrid convolutional neural network
MKC: Modified k-means clustering
RESNET: Residual neural network
TCIA: The cancer imaging archive
CLAHE: Contrast limited adaptive histogram equalization
ADF: Anisotropic diffusion filters
MSE: Mean squared error
HHO: Harris Hawks optimization
MCC: Matthews correlation coefficient.
